The article "The heterospin cobalt complexes: peculiarities of high-resolution NMR spectra" was published in 2022. Journal: Heliyon.

# The heterospin cobalt complexes: peculiarities of high-resolution NMR spectra

**DOI:** 10.1016/j.heliyon.2022.e09202

**Published:** 2022-03-31

**Authors:** V.K. Voronov, I.A. Ushakov, E.A. Funtikova

**Affiliations:** a Irkutsk National Research Technical University, Irkutsk, Russia; b A.E. Favorsky Irkutsk Institute of Chemistry, Siberian Branch, Russian Academy of Sciences, Irkutsk, Russia

**Keywords:** NMR, Paramagnetic shifts, Heterospin complexes

## Abstract

The high-resolution ^1^H and ^13^C NMR spectra (CHCl_3_ solution) of sterically non-rigid heterospin complexes CoL_2_, CoL_2_-dipy, and CoL_2_-phen (where L is 4-(3′,3′,3′-trifluoro-2′-oxopropylidene)-2,2,5,5-tetramethyl-3-imidazolidine-1-oxyl) have been studied. The specific of the NMR phenomenon in paramagnetic systems is briefly analyzed. It is shown that the NMR spectra modified by hyperfine coupling can be successfully employed for investigation of the complexation processes. In accordance with the common protocols, the ^1^H and ^13^C NMR signals are assigned using the information on ^13^С – ^1^Н spin-spin coupling. In addition, the preliminarily recorded ^1^H and ^13^C NMR spectra of radical L are also used in the work.

The temperature dependences of ^1^H and ^13^C paramagnetic shifts in the complexes under study have been obtained. A fundamental feature of these dependences is that they obey to the Curie law in a fairly wide temperature range (up to 100 °C). This observation can be used to control intramolecular processes of sterically nonrigid heterosystems in solutions.

## 1 Introduction

Currently, it is a common knowledge the phenomenon of nuclear magnetic resonance (NMR) in paramagnetic systems allows valuable (and often unique) information about the structure of matter to be obtained at the molecular level. This possibility is due to the electron-nuclear or hyperfine coupling (HFC) between unpaired electrons and resonating nuclei. Such a coupling dramatically transforms the NMR spectra, i.e. it induces paramagnetic chemical shifts of signals and their broadening. These features (with an appropriate analysis of such a transformation) permits to establish the peculiarities of spatial and electronic structure of multielectron (molecular) compounds (see, for example, reviews [1, 2, 3] and references cited therein). The real and wide possibilities of application of the HFC-modified NMR spectra were, for instance, summarized in the works [4, 5, 6]. These investigations have shown the efficiency of using the NMR phenomenon in paramagnetic complexes for addressing both research and applied tasks.

When it became possible to detect NMR spectra modified by hyperfine coupling, they started to be successfully employed for investigation of the complexation processes. This was demonstrated, for instance, by the study of molecular dynamics in solutions of transition metal paramagnetic ions with stable nitroxyl radicals, as well as by the investigation of intramolecular exchange and valence tautomerism in metal semiquinolates [7, 8]. In continuation of these researches, we have examined the ^1^H and ^13^С NMR spectra (in solution) of CoL_2_ (**1**), CoL_2_-dipy (**2**) and CoL_2_-phen (**3**) complexes (where L is 4-(3′,3′,3′-trifluoro-2′-oxopropylidene)-2,2,5,5-tetramethyl-3-imidazolidine-1-oxyl) (Scheme 1).

**Scheme 1:** Investigated complexes CoL_2_ (**1**), CoL_2_-dipy (**2**) and CoL_2_-phen (**3**), L is 4-(3′,3′,3′-trifluoro-2′-oxopropylidene)-2,2,5,5-tetramethyl-3-imidazolidine-1-oxyl).

According to the data of X-ray diffraction analysis, complexes **2** and **3** represent molecular structures. The similarity of elementary cells of **2** and **3** indicates isostructurality of the compounds. In each of them, the surrounding of metal atom is an octahedron with the *cis*-arrangement of paramagnetic ligands. The coordination sites of CoN_4_O_2_ fragment are formed by N and O atoms of the enaminoketone groups of two paramagnetic ligands and N atoms of bipyridyl or phenanthroline. The molecules of the complexes have axis pseudosymmetry of the second-order, which coincides with the bisector of NMN angle of the 5-membered chelate ring consisted of a metal atom with a diamagnetic ligand (Bipy or Phen). These chelate rings are practically planar, while 6-membered chelated metallocycles formed by a metal atom with a paramagnetic ligand have an inflection along the N…O bond with an angle of no more than 14.1° [9]. It is appropriate to note here that the interest of researchers in sterically non-rigid heterospin systems containing, in particular, radical fragments, as starting compounds for design of molecular magnets is still increasing (see, for example, [10]).

## 2 Analysis of NMR spectra of the complexes

Before analyzing the spectral information of complexes **1–3**, we have recorded the ^1^H and ^13^C NMR spectra of imidazolidine-1-oxyl ligand L. Due to the presence of a nitroxyl fragment in its molecule, the ^1^H NMR spectrum of this ligand is strongly broadened. In the spectrum, the main signals of 2- and 5-methyl groups with chemical shifts (XC, δ) are represented by broad lines with δ = -10.41 and -15.54 ppm, the signal of the olefinic proton H-6 has chemical shift of 7.72 ppm (Figure 1).

**Figure 1:** ^1^Н NMR spectrum of ligand L in СDCl_3_.

In accordance with the common protocols, the ^13^C NMR signals are assigned using the information on ^13^С – ^1^Н spin-spin coupling. However, very often the NMR signals in the spectra of paramagnetic compounds (in this case, of paramagnetic complexes) are so broadened due to HFC that this spin-spin coupling does not appear. Moreover, at sufficiently high values of HFC constants, the signals may not be detected at all [1].

The ^13^C NMR spectrum of radical L (Figure 2) gives the information, which allows the spectra of the studied complexes to be analyzed. This spectrum shows spin-spin coupling for two signals with chemical shifts (δ) of 107 and 172 ppm attributable to the carbon atoms of the CF_3_ group and C-7, respectively. The multiplicity of these signals is owing to the spin-spin coupling of ^13^C and ^19^F nuclei (JC−F1=290,8Hz,JC−F2=30,2Hz). It was previously reported [7] that the highest values of HFC constants for this compound (radical L) should be for carbons of СН_3_-groups, as well as for С-2 and С-5, which are most closely located to the paramagnetic site (N-oxyl fragment) in comparison with other carbon atoms. Therefore, because of a strong broadening, the signals of these carbons are absent in the spectrum shown in Figure 2. Thus, two other of four signals are due to the resonance of the C-4 and C-6 atoms. In this case, the high-field (most broadened) signal should be assigned to the C-4 atom, which, in terms of its location, should be more susceptible to the influence of the unpaired electron spin (by the contact and pseudo-contact mechanisms).

**Figure 2:** ^13^С NMR spectrum of radical L in СDCl_3_.

The C-4 atom upon coordination should be more affected by the uncompensated electron spin of the central ion of the paramagnetic complex (according to the σ-mechanism [1]) than the above three other carbon atoms. Such HFC should lead to a paramagnetic shift, as well as to even larger broadening of the signal up to its disappearance from the spectrum.

In the ^1^H NMR spectrum of complex 1, four broadened signals are observed (Figure 3). Basing on the integral intensities of the signals, the resonance with δ = -23.09 ppm can be assigned to a signal of H-6 proton of the imidazolidine fragment. Other signals have an intensity multiple of three: the signal with δ = -1.71 ppm corresponds to the common resonance of 5-CH_3_ group. In accordance with [11], signals with δ = -29.79 and -50.53 ppm are attributable to the methyl group proton in the position 2. A significant difference in the positions of signals of CH_3_ group protons is due to the effect of additional paramagnetic contribution (apart from the nitroxyl radical) on the protons of the methyl groups in position 2 of the cycle, closely located to the coordination center.

**Figure 3:** ^1^Н NMR spectrum of complex **1** in СDCl_3_.

The ^13^C NMR spectrum of complex **1** shows only three signals (Figure 4). Considering the ^13^C NMR spectrum of ligand L, it can be assumed that the signals with chemical shifts at 270, 396, and 479 ppm are due to the carbon atoms of CF_3_ group, C-6 and C-7, respectively. It should be additionally noted that significant broadenings in the ^1^H and ^13^C NMR spectra can be caused by the conformational mobility of the complex in a solution (Scheme 2) [7].

**Figure 4:** ^13^С NMR spectrum of complex **1** in СDCl_3_.

**Scheme 2:** Possible conformations of complex **1**.

The introduction of an additional chelate (2,2′-dipyridyl (*dipy*) or phenanthroline (*phen*)) fixes geometry of the complex and affects the position and width of signals in the NMR spectra.

The ^1^H NMR spectrum of complex **2** at room temperature contains a number of broadened signals in the region of δ = –45-35 ppm (Figure 5). The high-field signals have an integral intensity that is a multiple of three: they are assigned to the methyl groups in the positions 2 and 5 of the imidazolidine ring. Other signals belong to 2,2′-dipyridine and H-6 proton. In view of symmetry of the dipyridine ligand, the signal intensities are multiple of two.

**Figure 5:** ^1^Н NMR spectrum of complex **2** in СDCl_3_.

The ^13^C NMR spectrum for complex **2** also demonstrates high paramagnetic shifts for resonating carbon atoms. Taking into account the symmetry of the ligand (dipyridyl) and the presence of two ligands L, the spectrum should contain 15 signals, only 8 being detected (Figure 6). In the ^13^С NMR spectrum of complex 2, recorded without proton decoupling, only one doublet is detected at room temperature. However, the low-temperature experiments (T = 233 K and lower) reveal that the signals with chemical shifts at 219, 344, 454 ppm represent doublets with spin-spin coupling constants ^1^J(C, H) = 160 Hz that allows them to be assigned to the pyridine rings.

**Figure 6:** The ^13^С NMR spectrum without proton decoupling of complex **2** in СDCl_3_.

The ^1^H NMR spectrum of complex **3** at room temperature also shows significant paramagnetic shifts of the signals, which are so narrow that the signals of four methyl groups of ligand L appear as separate ones that can be integrated (Figure 7). This is explained by the fixation of octahedral geometry of the complex due to the introduction of phenanthroline. The ^13^C NMR spectrum of complex **3**, recorded without proton decoupling at room temperature, contains 4 doublets with constants ^1^J_СН_ ≈ 160 Hz (Figure 8). From possible 16 signals of the complex, only 9 signals are detected. Other signals are apparently strongly broadened due to the above reasons.

**Figure 7:** ^1^Н NMR spectrum of complex **3** in СDCl_3_.

**Figure 8:** ^13^С NMR complex of complex **3** in СDCl_3_ recorded without proton decoupling.

We have obtained the temperature dependences of paramagnetic shifts in the ^1^H and ^13^C NMR spectra of complexes **2** and **3** (Figures 9, 10, and 11). The numbering of the ligand atoms is shown in Scheme 3.

**Figure 9:** Temperature dependencies of chemical shifts in signals of methyl group protons of complexes **2** (а) and **3** (b) in the ^1^H NMR spectra.

**Figure 10:** Temperature dependencies of chemical shifts of aromatic protons in complexes **2** (а). and **3** (b) in the ^1^H NMR spectra.

**Figure 11:** Experimental dependencies ω(1/T) in the ^13^С NMR spectra of cobalt complexes **2** (а) and **3** (b).

**Scheme 3:** The numbering of ligand atoms in complexes CoL_2_-dipy (**2**) and CoL_2_-phen (**3**), L is 4-(3′,3′,3′-trifluoro-2′-oxopropylidene)-2,2,5,5-tetramethyl-3-imidazolidine-1-oxyl).

A fundamental feature of the above dependences is that they obey to the Curie law at a fairly wide temperature range (up to 100 °C). This experimental fact can be used to control the processes of intramolecular dynamics associated with the synthesis and study of sterically non-rigid heterosystems in solutions, including the design of molecular magnets.

## 3 Experimental

The ^1^H and ^13^C NMR spectra were recorded on a Bruker DPX250 pulse spectrometer in 5 mm ampoules using a BBO5mmZ3074/58 broadband probe. CDCl_3_ was used as a solvent. The values of chemical shifts in the ^1^H and ^13^C NMR spectra were recalculated relative to tetramethylsilane (TMS), which was used as an external standard. The concentrations of solutions for recording ^1^H and ^13^C NMR spectra were 5% and 10%, respectively. The ^1^H NMR spectra were recorded using the following parameters: spectral width 200 ppm, relaxation delay 1 s, number of scans 64. The ^13^C NMR spectra were recorded using the following parameters: spectral width 1500 ppm, relaxation delay 0.1 s, number of scans 30,000–50,000. The synthesis of the compounds studied by us is described in the work [9].

## 4 Conclusions

In conclusion, the ^1^H and ^13^C NMR spectra of CoL_2_ (**1**), CoL_2_-dipy (**2**) and CoL_2_-phen (**3**) complexes in solution have been studied. The assignment of NMR signals from carbon nuclei is based on the information used about the spin-spin interaction ^13^C – ^1^H. The initial information for such a reference was the parameters of the NMR spectrum previously obtained by us 4-(3′,3′,3′-trifluoro-2′-oxopropylidene)-2,2,5,5-tetramethyl-3-imidazolidine-1-oxyl. It is found that the paramagnetic shifts, induced in the NMR spectra of the cobalt complexes, obey to the Curie law in a fairly wide temperature range. Thus, the temperature dependences of paramagnetic shifts of NMR signals can be used to control intramolecular transformations in paramagnetic heterospin complexes in solutions. These dependencies make it possible to isolate solid phases of a certain structure from the solutions of such complexes.

The authors express their gratitude to Professor V.I. Ovcharenko for the compounds provided for the study.

## Declarations

### Author contribution statement

V.K. Voronov: Analyzed and interpreted the data; Wrote the paper.

I.A. Ushakov: Conceived and designed the experiments; Performed the experiments; Wrote the paper.

E.A. Funtikova: Contributed reagents, materials, analysis tools or data; Wrote the paper.

### Funding statement

This research did not receive any specific grant from funding agencies in the public, commercial, or not-for-profit sectors.

### Data availability statement

Data included in article/supplementary material/referenced in article.

### Declaration of interests statement

The authors declare no conflict of interest.

### Additional information

No additional information is available for this paper.
